The article "Influencing Factors of Daytime Sleepiness in Patients with Obstructive Sleep Apnea Hypopnea Syndrome and Its Correlation with Pulse Oxygen Decline Rate" was retracted in 2023. Reasons: suspected computer-generated content; unreliable results or conclusions; concerns about the data; concerns about the results or conclusions.

# Influencing Factors of Daytime Sleepiness in Patients with Obstructive Sleep Apnea Hypopnea Syndrome and Its Correlation with Pulse Oxygen Decline Rate

**DOI:** 10.1155/2021/6345734

**Published:** 2021-09-13

**Authors:** Fengying Zhang, Xijiang Wu, Wenping Duan, Fangfang Wang, Tingting Huang, Meiling Xiang

**Affiliations:** ^1^Department of Otorhinolaryngology, Weifang Hospital of Traditional Chinese Medicine, Weifang, Shandong 261041, China; ^2^Department of Otorhinolaryngology, Shouguang People's Hospital, Shouguang, Shandong 262700, China

## Abstract

**Objective:**

To explore the influencing factors of daytime sleepiness in patients with obstructive sleep apnea hypopnea syndrome (OSAHS) and the correlation between daytime sleepiness and pulse oxygen decline rate in patients with severe OSAHS.

**Methods:**

From January 2018 to April 2021, 246 consecutive patients with OSAHS diagnosed by polysomnography (PSG) in our hospital were selected. All patients were grouped according to the minimum nocturnal oxygen saturation and apnea hypopnea index (AHI). There were 33 cases in the no sleep hypoxia group, 34 cases in the mild hypoxia group, 119 cases in the moderate hypoxia group, and 60 cases in the severe hypoxia group. There were 30 cases in the simple snoring group, 55 cases in the mild OSAHS group, 48 cases in the moderate OSAHS group, and 113 cases in the severe OSAHS group. The Epworth Sleepiness Scale (ESS) scores of each group were compared. All patients were grouped according to ESS score. Those with score ≥9 were included in the lethargy group (*n* = 118), and those with score ≤10 were included in the no lethargy group (*n* = 128). Univariate and multivariate logistic regression analyses were used to explore the influencing factors of daytime sleepiness in OSAHS patients. Pearson correlation analysis showed the correlation between ESS score and pulse oxygen decline rate in patients with severe OSAHS.

**Results:**

The ESS score of the severe hypoxia group > the moderate hypoxia group > the mild hypoxia group > the no sleep hypoxia group. There was significant difference among the groups (*F* = 19.700, *P* < 0.0001). There were significant differences between the severe hypoxia group and other groups and between the moderate hypoxia group and the no sleep hypoxia group and the mild hypoxia group (*P* < 0.05). The ESS score of the severe OSAHS group > the moderate OSAHS group > the mild OSAHS group > the simple snoring group. There was significant difference among the groups (*F* = 19.000, *P* < 0.0001). There were significant differences between the severe OSAHS group and other groups and between the moderate OSAHS group and the simple snoring group (*P* < 0.05). Univariate analysis showed that BMI, neck circumference, snoring degree, total apnea hypopnea time, AHI, micro arousal index (MAI), oxygen saturation (CT90%), lowest oxygen saturation (LSaO2), and mean oxygen saturation (MSaO2) were the influencing factors of daytime sleepiness in OSAHS patients (*P* < 0.05). Multiple logistic regression analysis showed that AHI and CT90% were independent risk factors for daytime sleepiness in OSAHS patients (*P* < 0.05). Pearson correlation analysis showed that there was a positive correlation between ESS score and pulse oxygen decline rate in patients with severe OSAHS (*r* = 0.765, *P* < 0.0001).

**Conclusion:**

OSAHS patients may be accompanied by daytime sleepiness in varying degrees, which may be independently related to AHI and CT90%. The degree of daytime sleepiness in patients with severe OSAHS may be closely related to the decline rate of pulse oxygen, which should be paid great attention in clinic.

## 1. Introduction

Adult obstructive sleep apnea hypopnea syndrome (OSAHS) is a sleep disordered breathing disease in which patients are in a state of hypopnea or have apnea more than 30 times during continuous 7 h night sleep, or patients are in a state of hypopnea or have apnea more than 5 times/h [1]. The main clinical manifestations of this disease are excessive sleepiness, decreased memory and attention, even cognitive dysfunction or behavioral abnormalities in the daytime, irregular snoring and loud snoring, apnea, frequent hypoxemia caused by hypopnea, wakefulness, and sleep disorders during sleep at night [2, 3]. The affected patients vary widely, with single or multiple symptoms, or no symptoms at all. Existing studies have shown that OSAHS, as a systemic disease, is closely related to cardiovascular events such as hypertension, diabetes, coronary heart disease, arrhythmia, and heart failure, and its consequences also include increased risks of sudden death, work-related accidents, and traffic accidents caused by sleep disorders and cardiovascular events [4–6]. Clinical examination and a typical history are used to diagnose the disease. According to relevant statistics, body mass index (BMI) ≥ 28 kg/m^2^, age increase, menopause, upper airway anatomical structure abnormalities, long-term smoking, long-term heavy drinking, and family history of OSAHS are all important inducers or risk factors for OSAHS [7, 8]. Recent studies have also shown that long-term chronic hypoxia is an important mechanism leading to daytime sleepiness, and repeated intermittent hypoxemia at night is the main determinant of daytime sleepiness in OSAHS patients, and for some OSAHS patients with severe obstructive apnea, arterial oxygen saturation is low when they are awake, therefore, daytime sleepiness with higher performance [9, 10]. At present, studies on the correlation between nocturnal intermittent hypoxia and daytime sleepiness in OSAHS mostly focus on the severity, duration, and frequency of hypoxia. Pulse oxygen decline rate is an important parameter reflecting the severity of hypoxemia, which represents the rate of deoxygenation saturation during apnea. Research [11] shows that when apnea occurs, the rapidly decreasing blood oxygen saturation can easily lead to serious mismatch of ventilation and blood perfusion ratio and lead to multiple organ injury. Based on this, it is of great clinical value to study the influencing factors of daytime sleepiness and its correlation with nocturnal hypoxemia in patients with OSAHS, and as a new sleep monitoring index, pulse oxygen decline rate should receive more attention. This study explored the influencing factors of daytime sleepiness in patients with OSAHS and further explored the correlation between pulse oxygen decline rate and daytime sleepiness in patients with severe OSAHS. See the report for details.

## 2. Materials and Methods

### 2.1. General Data

From January 2018 to April 2021, 246 consecutive patients who underwent polysomnography (PSG) and were diagnosed as OSAHS in our hospital were selected. The diagnostic criteria of OSAHS and the disease classification of nocturnal minimum oxygen saturation and apnea-hypopnea index (AHI) referred to the international classification of sleep disorders [12]. See Table 1 for details.

### 2.2. Inclusion Criteria

Patients accompanied by sleepiness, snoring, dry mouth, and other symptoms; aged 18–70 years old; with blood pressure <180/110 mmHg; with AHI > 5 times/h; with normal self-care ability and cognitive function; and with PSG monitoring signal integrity were included.

### 2.3. Exclusion Criteria

Patients combined with narcolepsy or insomnia; complicated with serious or unstable basic medical diseases; complicated with mental disorders; and with long-term use history of sedatives and antidepressants and recent use history of excitatory drugs and patients with cerebrovascular diseases such as head injury, epilepsy, intracerebral hemorrhage, cerebral thrombosis, and brain tumor and complicated with infection and metabolic poisoning were excluded.

### 2.4. Research Methods and Observation Indexes

All patients were monitored with German somno multichannel sleep monitor for more than 7 h at night. The observation indexes included total apnea hypopnea time, maximum apnea time, AHI, micro arousal index (MAI), oxygen saturation (CT90%), minimum blood oxygen saturation (LSaO_2_), and mean blood oxygen saturation (MSaO_2_). The data analysis was completed according to the OSAS diagnosis and treatment guidelines of the American Academy of Sleep Medicine [13]. All patients were grouped according to the minimum nocturnal oxygen saturation and AHI. There were 33 cases in the no sleep hypoxia group, 34 cases in the mild hypoxia group, 119 cases in the moderate hypoxia group, and 60 cases in the severe hypoxia group. There were 30 cases in the simple snoring group, 55 cases in the mild OSAHS group, 48 cases in the moderate OSAHS group, and 113 cases in the severe OSAHS group. The Epworth Sleepiness Scale (ESS) scores of each group were compared. All patients were grouped according to ESS score. Those with score >10 were included in the lethargy group (*n* = 118)/47.97%, and those with score ≤10 were included the no lethargy group (*n* = 128)/52.03%. The general information of all patients was collected, and the influencing factors of daytime sleepiness in OSAHS patients were discussed by univariate and multivariate logistic regression analysis. Pearson correlation analysis showed the correlation between daytime sleepiness and nocturnal hypoxemia (ESS score and pulse oxygen decline rate) in patients with severe OSAHS. Analysis of pulse oxygen decline rate: the time from the starting point of blood oxygen saturation decline to its lowest point was calculated as Δ*t*. The amplitude of pulse oxygen decrease at this time point was ΔSpO2_∘_ΔSpO2/Δ*t* (%/s); it was used to represent the desaturation rate per unit time, which is the pulse oxygen decline rate [14].

### 2.5. Statistical Methods

SPSS22.0 software was used for processing. All measurement data were in accordance with normal distribution, expressed in ($\bar{x}$ ± *s*), analysis of variance was used for intergroup comparison, and *t*-test was used for pairwise comparison. Categorical variable data and descriptive analysis were expressed in (%) and implemented *χ*^2^ inspection. The significant factors in univariate analysis were analyzed by multiple logistic regression model. Pearson correlation analysis was used for correlation analysis. When *P* < 0.05, there was significant difference between them.

## 3. Results

### 3.1. Comparison of ESS Scores in Each Group

The ESS score of the severe hypoxia group > the moderate hypoxia group > the mild hypoxia group > the no sleep hypoxia group. There was significant difference among the groups (*F* = 19.700, *P* < 0.0001). There were significant differences between the severe hypoxia group and other groups and between the moderate hypoxia group and the no sleep hypoxia group and the mild hypoxia group (*P* < 0.05). The ESS score of the severe OSAHS group > the moderate OSAHS group > the mild OSAHS group > the simple snoring group. There was significant difference among the groups (*F* = 19.000, *P* < 0.0001). There were significant differences between the severe OSAHS group and other groups and between the moderate OSAHS group and the simple snoring group (*P* < 0.05), as seen in Figure 1.

### 3.2. Univariate Analysis of Daytime Sleepiness in OSAHS Patients

The results showed that BMI, neck circumference, snoring degree, total apnea hypopnea time, AHI, MAI, CT90%, LSaO_2,_ and MSaO_2_ were the influencing factors of daytime sleepiness in OSAHS patients (*P* < 0.05), as seen in Table 2.

### 3.3. Multiple Logistic Regression Analysis of Daytime Sleepiness in OSAHS Patients

The results showed that AHI and CT90% were independent risk factors of daytime sleepiness in OSAHS patients (*P* < 0.05), as seen in Tables 3–4.

### 3.4. Correlation Analysis between ESS Score and Pulse Oxygen Decline Rate in 113 Patients with Severe OSAHS

Pearson correlation analysis showed that there was a positive correlation between ESS score and pulse oxygen decline rate in patients with severe OSAHS (*r* = 0.765, *P* < 0.0001), as seen in Figure 2.

## 4. Discussion

Daytime sleepiness refers to patients' uncontrollable sleep tendency during the day. Its incidence is high in OSAHS patients, up to 30.9–69.3%, which has an adverse impact on patients' spirit, cognitive function, quality of life, and work efficiency [15]. In this study, the incidence of daytime sleepiness was 47.97%, nearly half. It can be seen that daytime sleepiness is widespread and harmful in patients with OSAHS, which should be paid attention to clinically.

The mechanism of daytime sleepiness in OSAHS patients is not clear. At present, it is generally believed that it is related to sleep fragmentation and nocturnal hypoxemia, which can also be independent risk factors [16]. The main manifestations were obvious nocturnal hypoxia in tissue, shortened sleep latency, and improved sleep efficiency. Nocturnal minimum oxygen saturation and AHI are two important indexes to evaluate the severity of OSAHS; ESS is an important tool for self-assessment of daytime sleepiness in patients with OSAHS [17]. In the results of this study, the ESS score of the severe hypoxia group > the moderate hypoxia group > the mild hypoxia group > the no sleep hypoxia group. There was significant difference among the groups. There were significant differences between the severe hypoxia group and other groups and between the moderate hypoxia group and the no sleep hypoxia group and the mild hypoxia group. The ESS score of the severe OSAHS group > the moderate OSAHS group > the mild OSAHS group > the simple snoring group. There was significant difference among the groups. There were significant differences between the severe OSAHS group and other groups and between the moderate OSAHS group and the simple snoring group. It is suggested that the ESS score of OSAHS patients increases with the severity of the disease, that is, the decrease of nocturnal minimum oxygen saturation and the increase of AHI.

The present study found that BMI and excessive daytime sleepiness were positively correlated with the severity of OSAHS, and low blood oxygen, respiratory disturbance index, micro arousal index, and the longest/average duration of sleep breathing were all related to the daytime sleepiness of patients [18]. In the study, univariate analysis showed that BMI, neck circumference, snoring degree, total apnea hypopnea time, AHI, MAI, CT90%, LSaO_2_, and MSaO_2_ were the influencing factors of daytime sleepiness in OSAHS patients. It was partially consistent with the above research. It was suggested that the abovementioned factors and ESS evaluation tools could be used as the preliminary diagnosis basis of daytime sleepiness in OSAHS patients. Previous studies had also found that obesity was related to sleepiness, and its mechanism might be related to obesity-derived factors (tumor necrosis factor, interleukin-6, etc.) [19]. This study found that the proportion of men and women with OSAHS and OSAHS daytime sleepiness was much higher in men than in women. We analyzed the reasons as follows: Compared with women, men are more prone to airway stenosis due to a large amount of fat deposition in the palatopharyngeal plane and a large amount of neck soft tissue. In addition, male hormone testosterone can also aggravate sleep apnea [20]. Snoring is one of the important manifestations of OSAHS patients, which can cause soft tissue vibration. This study found that the heavier the degree of snoring, the greater the possibility of daytime sleepiness, suggesting that the degree of snoring is related to daytime sleepiness. Total apnea hypopnea time can reflect the authenticity of apnea time and occurrence times of OSAHS patients during all night sleep, AHI can reflect the times of apnea of OSAHS patients, and MAI can reflect the times of micro awakening of OSAHS patients. The higher the three indexes, the worse the sleep continuity and sleep quality, so it can cause daytime sleepiness symptoms of patients. CT90%, LSaO_2_, and MSaO_2_ are related indicators of oxygen saturation. In the study, the CT90% of the lethargic group was higher than that of the no lethargic group, and the LSaO_2_ and MSaO2 were lower than that of the no lethargic group, which confirmed the previous study's argument that hypoxemia was closely related to daytime sleepiness [21]. The reasons were analyzed, which may be related to the damage of cerebral cortical neurons caused by systemic inflammation and oxidative stress induced by hypoxemia [22]. In the study, multiple logistic regression analysis showed that AHI and CT90% were independent risk factors for daytime sleepiness in OSAHS patients. However, some scholars believe that AHI is not strongly correlated with the degree of daytime sleepiness in patients with OSAHS, and its decisive factor is mainly nocturnal hypoxemia, and the heavier its degree is, the stronger its correlation with ESS score [23]. This suggests that compared with simple oxygen saturation index and AHI, CT90% can better reflect the possibility of daytime sleepiness in OSAHS patients. Therefore, in the clinical diagnosis and treatment of OSAHS patients with low ESS score, more emphasis should be placed on the monitoring and analysis of CT90%, so as to reduce the missed diagnosis rate and reduce the risk. ESS score can reflect the severity of daytime sleepiness in patients with OSAHS, and the decrease rate of pulse oxygen can reflect the oxygen reduction events after nocturnal apnea. Existing studies have shown that the decrease rate of pulse oxygen is significantly correlated with AHI, and the reason why OSAHS patients with similar AHI differ in their daytime sleepiness is related to the decrease rate of pulse oxygen. In the study, Pearson correlation analysis showed that there was a positive correlation between ESS score and pulse oxygen decline rate in patients with severe OSAHS. It is suggested that the increase of pulse oxygen decline rate can lead to the aggravation of daytime sleepiness in patients with severe OSAHS, which is consistent with the above research point of view. The reasons were analyzed. After apnea, the pulse oxygen decline rate is mainly affected by oxygen reserve (this is the residual capacity of lung function); when oxygen reserve is insufficient, the body is hypoxic, the patient's oxidative stress is enhanced, the inflammatory level is increased, and the neurons in cerebral cortex are damaged, which can lead to sleepiness symptoms [24]. In addition, the decrease of residual capacity of pulmonary function is directly proportional to obesity, and the inflammatory factors derived from obesity may have a synergistic effect combined with it [25].

In conclusion, OSAHS patients may be accompanied by daytime sleepiness in varying degrees, which may be independently related to AHI and CT90%. The degree of daytime sleepiness in patients with severe OSAHS may be closely related to the decline rate of pulse oxygen, which should be paid great attention in clinic.

## Figures and Tables

**Figure 1:** Comparison of ESS scores in each group ($\bar{x}$ ± *s*, points). (a) The ESS score of OSAHS patients with different degrees of hypoxia at night. The ESS scores of the no sleep hypoxia group, mild hypoxia group, moderate hypoxia group, and severe hypoxia group were (6.15 ± 2.76), (7.21 ± 3.58), (9.92 ± 4.62), and (13.71 ± 7.46) points, respectively. (b) The ESS scores of OSAHS patients with different severity. The ESS scores of the simple snoring group, mild OSAHS group, moderate OSAHS group, and severe OSAHS group were (5.97 ± 3.10), (6.88 ± 3.91), (8.47 ± 4.69), and (12.25 ± 6.61) points, respectively. ^*∗*^stands for comparison with the no sleep hypoxia group and simple snoring group, *P* < 0.05; ^#^stands for comparison with the mild hypoxia group and mild OSAHS group, *P* < 0.05; ∆ stands for comparison with the moderate hypoxia group and moderate OSAHS group, *P* < 0.05.

**Figure 2:** Scatter plot of correlation between ESS score and pulse oxygen decline rate in 113 patients with severe OSAHS.

**Table 1:** Severity of OSAHS in adults.

Degree	Minimum oxygen saturation at night (%)	AHI (times/h)
Mild	85–90	5–15
Moderate	80 ∼< 85	>15–30
Severe	<80	>30

**Table 2:** Univariate analysis of daytime sleepiness in OSAHS patients.

Factors	Lethargy group (*n* = 118)	No lethargy group (*n* = 128)	*χ*^*2*^/*t*	*P* value
Gender (cases)			0.049	0.826
Male	107	115		
Female	11	13		
Age (years old)	41.69 ± 5.34	42.02 ± 5.27	0.488	0.626
BMI (kg/m^2^)	28.45 ± 4.19	27.14 ± 2.56	2.985	0.003
Neck circumference (cm)	42.84 ± 3.38	41.61 ± 3.45	2.821	0.005
Degree of snoring (cases)			11.730	0.003
Mild	11	27		
Moderate	15	27		
Severe	92	74		
Total apnea hypopnea time (min)	143.14 ± 73.61	91.40 ± 76.57	5.394	<0.001
Maximum apnea time (s)	62.36 ± 19.60	57.29 ± 20.84	1.961	0.051
AHI (times/h)	49.85 ± 21.66	37.52 ± 23.10	4.309	<0.001
MAI (/h)	36.27 ± 19.94	26.68 ± 18.17	3.947	<0.001
CT90% (%)	26.28 ± 24.03	8.42 ± 10.44	7.662	<0.001
LSaO_2_ (%)	66.21 ± 18.25	74.22 ± 10.65	4.244	<0.001
MSaO_2_ (%)	90.34 ± 5.87	94.16 ± 2.43	6.762	<0.001

**Table 3:** Assignment for multivariate analysis of factors.

Factors	Variables	Assignment
AHI	*X*1	Normal = 0, 5–15 (times/h) = 1, >15–30 (times/h) = 2, >30 (times/h) = 3
CT90%	*X*2	>90% = 0, ≤90% = 1

**Table 4:** Multiple logistic regression analysis of daytime sleepiness in OSAHS patients.

Factors	*β*	SE	Wald	*P* value	OR (95% CI)
AHI	0.774	0.375	4.428	0.023	2.184 (1.058 – 4.425)
CT90%	1.473	0.474	9.747	0.003	4.365 (1.733 – 11.010)

## Data Availability

The primary data used to support the results of this study are available from the corresponding author upon reasonable request.
